The article "Green Message Framing in Enhancing Sustainable Consumption Behavior of Fashion Based on the Cross-Theoretical Model" was published in 2022. Journal: J Environ Public Health.

# Green Message Framing in Enhancing Sustainable Consumption Behavior of Fashion Based on the Cross-Theoretical Model

**DOI:** 10.1155/2022/4038992

**Published:** 2022-09-05

**Authors:** Lihong Chen, Lin He, Xinfeng Yan, Chunhong Liu

**Affiliations:** ^1^Shanghai International Fashion Science and Innovation Center, Donghua University, Shanghai 200051, China; ^2^Glorious Sun School of Business and Management, Donghua University, Shanghai 200051, China; ^3^International Cultural Exchange School, Donghua University, Shanghai 200051, China

## Abstract

Promoting green consumption is key in meeting ambitious sustainable fashion targets being set around the world. This research examined how framing of green message as positive or negative (i.e., benefit framing) influenced formation of sustainable consumption behaviors of fashion (SCBF) based on the cross-theoretical model and, especially, how self-efficacy, decision balancing, and perceiving threats-mediated green message framing effects. Data were collected from 217 Chinese residents in an online experiment. Our findings show that green message framing has different effects on individuals in different change stages of SCBF and loss framing-based green messages induce more positive responses toward SCBF with greater perceived threats in the pre-intention and intention stages, while gain framing-based green messages might stimulate positive behaviors toward SCBF with greater perceived benefits in the preparation and action and maintenance stages. Results suggest that highlighting green message expression in relating to SCBF may be useful for promoting broader sustainable behaviors. Therefore, this article significantly fills the gaps between green message framing and SCBF. The findings of this article have significant implications for fashion companies who wish to explore the fashion green market potential.

## 1. Introduction

Growing concerns over climate change and environmental issues are making governments and citizen groups attentive to changing the way people consume on fashion [1]. As early as 1992, the United Nations Conference on Environment and Development had pointed out that consumer behavior was closely related to environmental issues. Anticipating continued increased attention from consumers on sustainability issues, considerable attention has been directed toward sustainable consumption behaviors of fashion (SCBF) intended to reduce negative environmental harm [2]. In this regard, scholars and public policy makers stress the urgency to motivate consumers to engage in SCBF; the relevant enterprises and organizations have taken many publicity measures to convey green messages and promote the sustainable consumption of fashion [3–5]. However, due to the neglect of the important role of expression of green messages and consumer demand in the dissemination of green messages, many education and publicity effects are not ideal, and there is still a gap between consumers' intention and behavior to consume sustainable fashion. What kind of green messages can arouse consumer recognition more? How should green messages be delivered in order to effectively promote the formation of SCBF? These issues deserve our further attention and research.

Furthermore, despite a diverse array of green messages designed to direct at individuals to care about the environment and save resources [6, 7], it is unclear how many customers carefully read and internalize such messages, what type of green messages have the greatest effect upon consumers, and how likely they are to change their SCBF in keeping with those messages. Researchers have verified the effectiveness of green messages on sustainable consumption behavior [8] and have increasingly focused on the expression of green messages, namely, the effect of green message frame [9]. Previous researches involved the impact of green message framing on individual environmental behavior, energy-saving behavior, water-saving behavior, green travel, greenhouse gas emissions, and the purchase of green products [9–13]. However, few studies have investigated the effects of green message framing in terms of SCBF.

A great deal of research has been devoted to examining how individual perceptions are affected by message framing as a guide to constructing appropriate messages [14]. Message framing can be used to focus on individual's attention on some aspect of the message [9]. In green message framing, the message is framed so as to make an individual feel gain or loss; such green messages would thus relate to consumer decision making [10]. The provision of green message can be seen as an expression to increase the likelihood of intention or behavior of sustainable consumption. With regard to expression of green messages, it is noted that positive or negative expression affects how green messages are perceived and their impact on consumers' intention and behaviors toward sustainable fashion consumption [6]. Appropriate expression of green messages is an essential tool for individuals to change their perception and behaviors. Therefore, this article frames the gain and loss framing of green messages, aims to explore the influencing mechanism of green message framing on SCBF, and provides suggestions for enterprises to carry out more targeted green marketing.

Lastly, it can be seen that consumers' awareness of SCBF is gradually increasing, but the behavior formation is not good. Existing studies in sustainable consumption behavior have examined the influencing attributes based on planned behavior theory, value-belief-norm theory, and interpersonal relationship theory [15, 16], which consider sustainable consumption behavior as a static status and cannot well explain the differences of “intention-behavior.” Therefore, aiming at the appeal problem, this article introduces the transtheoretical model into the field of SCBF, combines the framing message with the transtheoretical model, and studies the impact of the gain and loss framing-based green messages on the “intention-behavior” formation process in SCFB of individuals.

Taken together, this research provides policy makers and business strategists with useful insights to cultivate and drive SCBF, design green messages, and accurately present green message to consumers to facilitate the consumer formation of SCBF. This is achieved by analyzing the relationship between the gain and loss framing, self-efficacy, decision balancing, perceived threats, and the change stages of SCBF based on the cross-theoretical model, which explores the influence mechanism of green message framing on SCBF. To this end, research hypotheses are proposed and justified in the following section. Next, the research methods and empirical results are described. The last section draws implications for theory and practice.

## 2. Hypotheses Development

### 2.1. Green Information Framing and Sustainable Consumption Behavior of Fashion

Previous research shows that how green message is presented can significantly promote individuals' willingness and action to participate in environmentally friendly behaviors, which means that appropriate message framing can improve the persuasiveness of green message [17]. However, it is still uncertain whether gain framing or loss framing is better in encouraging consumers' sustainable consumption behavior [18]. On the one hand, some scholars believe that, for sustainable consumption behaviors or pro-environmental behaviors, gain message can more arouse positive emotions of individuals than loss message, by conveying the contribution of sustainable consumption to individuals or the environment, so that they are willing to make efforts for social, environmental, and personal interests. Gain message framing is more likely to promote consumer participation in energy-saving behaviors [19], stimulate individual green buying behaviors, attract individual attention to air pollution problems, and promote preventive measures and environmental behaviors than loss message framing. On the other hand, some scholars believe that loss message framing describes the harm caused by bad behavior to personal health and natural environment, which can better attract the attention of individuals and make them feel threatened, so that they are willing to change bad behavior to avoid harm. Loss message framing is more likely to promote consumer participation in hotel linen recycling projects [20], promote citizens' awareness of water conservation and water-saving behaviors in environmental public service advertisements, be conducive to individual choice of sustainable transportation in the study of the impact of transport CO_2_ emissions information on individual transportation choices [12], and be conducive to consumer use of eco-friendly biofuels when the negative impact of gasoline is emphasized [14].

According to prospect theory, people usually weigh their gains against losses before making decisions. When the gains in the situation are more obvious, people usually tend to be risk-averse, choosing profitable behaviors in order to maintain or enhance existing gains; when the loss is more obvious, people are often more inclined to identify risk in order to change the status, choosing behaviors that are likely to gain more. In this study, the individuals in the pre-intention stage and intention stage of SCBF are still in the early stages of behavior change, and there is no actual behavior change. Therefore, it is considered that sustainable consumption of fashion is a risk behavior for those consumers. Simultaneously, the loss message can better indicate that they are currently in a state of loss because they may concern personal or environmental harm caused by the unsustainable consumption of fashion. In the preparation and action and maintenance stages, consumers are gradually beginning to change behavior because the regression of the behavior stage is seen as a risk behavior. Meantime, because they are enjoying the benefits of sustainable consumption of fashion to individuals and environment, gain message framing can better strengthen the awareness of the benefits of their own state so as to promote them to avoid risks and continue to maintain or advance the formation of SCBF. Therefore, we propose the following hypotheses:

' *H1*. Loss framing based on a green message promotes consumers' formation of SCBF in the pre-intention and intention phases
 
*H2*. Gain framing based on a green message promotes consumers' formation of SCBF in the preparation and action and maintenance phases

### 2.2. Self-Efficacy

Self-efficacy mediates individual acquisition of knowledge, experience, and behavior [21]. It has been established as one of the most important mediators in gain and loss message framing studies [22]. Self-efficacy refers to the amount of confidence on whether they have sufficient ability to accomplish their target behavior [23]. As the executing agent of behavior, the successful execution of behavior depends to some extent on people's belief that they can achieve the goal [24]. The higher the self-efficacy of the individual, the higher the self-confidence of the individual in behavior change, the more the confidence in overcoming difficulties to complete the behavior change, the greater the possibility of changing behavior [21]. Obviously, individual choices and persistence in behavior are influenced by self-efficacy [23]. The mediating role of self-efficacy in message framing research has been greatly demonstrated in the studies of healthy behaviors. Self-efficacy is established to play a mediating role in message framing and human papillomavirus vaccine [25]. Gain message increases individual self-efficacy in physical activities more than loss message, thereby increasing the user's intention to use the fitness app [26]. Gain framing can promote the improvement of individual self-efficacy and thus promote the formation of individual healthy behaviors than loss framing [27]. In the studies on sustainable consumption behavior, researchers have also found that gain framing improves the public's self-efficacy more than loss framing, and individuals who believe they can promote sustainable consumption through action are more likely to engage in and maintain sustainable consumption behaviors than individuals who question their ability to conduct sustainable consumption [28]. Gain message can improve consumers' self-efficacy and thus promote the formation of sustainable consumption behaviors [29]. Morton noted that gain message can promote an individual's environmentally friendly behavior by stimulating an individual's self-efficacy [22]. Therefore, for SCBF, gain framing based on green message describes the benefits of sustainable consumption of fashion to individuals and the environment, enabling individuals to acquire the knowledge and skills of sustainable consumption of fashion and to believe that they can cope with the difficulties that may exist in sustainable consumption of fashion, so as to implement or adhere to sustainable consumption of fashion. Based on the above studies, the following hypotheses are suggested:

 
*H3a*. Gain farming based on a green message positively impacts self-efficacy in the preparation stage
 
*H3b*. Gain framing based on a green message positively impacts self-efficacy in the action and maintenance stage
 
*H4a*. Self-efficacy is positively associated with consumers' formation of SCBF in the preparation stage
 
*H4b*. Self-efficacy is positively associated with consumers' formation of SCBF in the preparation and action and maintenance stages
 
*H5a*. Self-efficacy mediates the relationship between gaining framing-based green messages and consumers' formation of SCBF in the preparation stage
 
*H5b*. Self-efficacy mediates the relationship between gaining framing-based green messages and consumers' formation of SCBF in the action and maintenance stage

### 2.3. Decision Balancing

Decision balance is the important variable to explain individual behavior change, including perceived benefit and perceptual barriers. Perceived benefit refers to the individual's perception on the benefits brought by behavior change, while perceptual barriers refer to the individual's perception on the obstacles or costs that may be encountered in the process of changing behavior [30]. Changes in individual behavior are caused through weighing perceived benefits against perceptual impairments, which promote behavioral changes, while perceptual impairment inhibits behavioral changes [31]. People always want to pay the least cost to reap the greatest benefits when making decisions, and people will only make decisions when the benefits obtained are greater than the costs [32]. Similarly, the implementation of sustainable consumption behavior depends on the weighing of the individual's trade-off of the costs to be paid and the benefits that can be obtained, and when people perceive that the benefits of sustainable consumption behavior are much higher than the costs, the bad behavior will be changed for personal gain. For example, people first consider the benefits of green products to the environment and personal health, as well as the difficulties caused by the higher price of green products before buying green products, and they will buy green products when the perception on the benefits of green products is greater than the obstacle to purchasing it [33]. In this study, because there are no obstacles and costs that need to be paid for the sustainable consumption of fashion, consumers' perception on sustainable consumption in fashion has basically not changed during the four changing stages. Therefore, the formation of consumers' SCBF is mainly due to the improvement of perceived benefits rather than the decline of perceptual barriers [32]. Gain message mainly describes the benefits of behavioral change, so perceived benefits are often mediated in the impact on behavioral change in message framing-related research. Gain framing based on advertising messages promotes consumers' perception on health and environmental benefits, making them more willing to buy organic foods [34]. Gain framing message can more effectively influence the perceived benefits of individuals than the loss framing messages, thereby promoting individual willingness of vaccination [35]. Gain framing message can also better promote individual participation in sports with perceived benefits acting as intermediaries [36]. In this study, gain framing based on green message involves the benefits of SCBF to individuals and the environment, so individuals will be more willing to adopt sustainable consumption behaviors of fashion when the perceived benefits are greater than the costs they need to pay. Based on the above studies, the following hypotheses are suggested:

 
*H6*. Perceived barriers are not associated with consumers' formation of SCBF
 
*H7a*. Gain framing-based green messages have a favorable impact on perceived benefits in the preparation stage
 
*H7b*. Gain framing-based green messages will have a favorable impact on perceived benefits in the action and maintenance stage
 
*H8a*. Perceived benefits are positively associated with consumers' formation of SCBF in the pre-intention phase
 
*H8b*. Perceived benefits are positively associated with consumers' formation of SCBF in the action and maintenance stage
 
*H9a*. Perceived benefits mediate the relationship between the gain framing-based green messages and consumers' formation of SCBF in the preparation stage
 
*H9b*. Perceived benefits mediate the relationship between the gain framing-based green messages and consumers' formation of SCBF in the action and maintenance stage

### 2.4. Perceived Threats

Perceived threats are individual's perception on the degree of harm caused by the external environment to himself, which are aroused by the appeal of fear. Perception on the level of threats will affect the individual's probability of adopting the recommended scenario. Loss message describes the harm of bad behavior, which can produce negative emotions such as fear and threat, and these negative emotions can make individuals tend to avoid bad behavior so that loss framing message can be effective in discouraging bad behavior [37]. The mediating role of perceived threats in message framing has been demonstrated in the research on healthy behaviors. Loss message is found to make individuals in grief more easily develop a sense of threat and behavior in the research on genital herpes message seeking [38]. Loss framing message is more persuasive than gain framing message when the object of message description is considered a threat [37]. Loss message describing that it will cause health problems affects an individual's perceived threat and perceived severity, prompting individuals to support weight loss policies [39]. Loss message describing the threats that smoking behavior poses to human health would make individuals feel frightened, thereby increasing the persuasiveness of the message [40]. When given a message about the negative effects of skin cancer on the appearance of the skin, people are more likely to feel the huge threat posed by skin cancer and are more willing to take skin protective behaviors [41]. In the research of sustainable consumption, when individuals realized the adverse effects of a certain behavior on their health and the ecological environment through loss message, the individual perceived threat will increase, which will cause the likelihood and severity of the perceived harm to continue to increase [42]. Furthermore, when it is felt that environmental problems have seriously affected the health and living environment of the individuals, they will not allow it to continue to develop and they will be motivated to deal with the threat [43]. In this research, loss framing-based green message conveys the damage of unsustainable consumption behavior of fashion to personal health and ecological environment, which is more likely to arouse people's attention to the problem of unsustainable consumption of fashion, enhance the recognition of the serious destruction, and thus seriously reflect on their current behavior. When the perceived threat is increasing, individuals will be more strongly aware of the harm caused by unsustainable consumption of fashion to the physical health of individuals and the bad situation of life, and they will make behavioral changes and adopt sustainable fashion consumption behaviors in order to avoid harm and change the status [33]. Based on the above studies, the following hypotheses are suggested:

 
*H10a*. Loss framing-based green messages have a favorable impact on a perceived threat in the pre-intention phase
 
*H10b*. Loss framing-based green messages have a favorable impact on a perceived threat in the intention phase
 
*H11a*. Perceived threats are positively associated with consumers' formation of SCBF in the pre-intention phase
 
*H11b*. Perceived threats are positively associated with consumers' formation of SCBF in the intention phase
 
*H12a*. Perceived threats mediate the relationship between the loss framing-based green messages and consumers' formation of SCBF in the pre-intention phase
 
*H12b*. Perceived threats mediate the relationship between the gain framing-based green messages and consumers' formation of SCBF in the intention phase

In the following section, green message framing, self-efficacy, decision balancing, perceiving threats, and fashion-sustainable consumption behavior are tested in a unified framework to gauge their respective associations with the formation of SCBF. Please refer to Figure 1.

## 3. Survey Experiments

### 3.1. Survey Experiment Design

This study employed survey experimental design, in which the phase of consumers' sustainable fashion consumption was investigated before and after the framing-based green message intervention. The survey experiments are divided into three parts, including pretest, green message intervention after the gain/loss framing, and posttest. The pretest questionnaire was designed to survey the phase of sustainable fashion consumption of participants before receiving green messages. Then a green message frame that was either gain or loss was designed as intervention material to conduct group intervention for participants. Furthermore, the posttest survey was used to investigate the phase of sustainable fashion consumption of participants after receiving green messages, which can be compared with the results of pretest so as to explore the different effects of gain/loss framing green messages. The experiments were conducted online, with pretest and posttest questionnaires distributed through “Questionnaire Star” software and intervention messages disseminated to participants through “WeChat” social platform.

Participants were first asked to watch a brief video about what is SCBF. Respondents completed a pretest questionnaire that measured the current status of SCBF. Subsequently, they were divided into four groups including pre-intention, intention, preparation, and action and maintenance according to the stage of SCBF of pretest subjects, and each group was randomly and uniformly divided into three groups to receive gain framing message, loss framing message and blank message intervention for one month (30 days). As the respondents deepened their understanding of sustainable fashion consumption behavior, the message intervention frequency was slowly extended from 2 days at a time, and a total of 9 interventions were conducted, and the specific intervention time is shown in Table 1. Among them, the gain framing group received the positive green messages, the loss framing group received the negative green messages, and the blank control group did not receive messages. Respondents answered a question related to the message materials after each message was distributed to ensure that they carefully read the messages; then they were asked to fill out the posttest questionnaire to measure the SCBF after the message intervention.

### 3.2. Questionnaire and Materials

The questionnaire consisted of three parts which were administered in a particular order. The first part investigated the sociodemographic characteristics. In the second part, the respondents had to read a message and answer questions relating to perceived self-efficacy, decision-making balance, and perceived threats of the messages. The third part investigated the change stage of SCBF in which respondents are. The pretest and posttest questionnaires were identical, except the framing of the green message the respondents had to read. The manipulation test scale is added to the posttest questionnaire to ensure that the experimental materials are clearly framed and the group intervention is successful, and the respondents in both the gain group and the loss group should answer one question.

Experimental stimulus materials are divided into two groups: the gain framing-based green messages and the loss framing-based green messages. The gain framing-based green messages emphasize the benefits of SCBF for individuals and the environment, while the loss framing-based green messages emphasize the harm to individuals and the environment caused by loss framing-based green messages. Two versions of green messages contain the same content. These benefits and hazards involve air quality, natural environment, living environment, resources, life and health, personal welfare, etc. The experimental materials include a total of 9 pairs and 18 articles, and each time a pair of materials is sent to the gain group and the loss group, the respondents are required to answer a simple reading comprehension question related to the materials.

### 3.3. Participants

Responses were collected from 217 Chinese residents in the pretest experiment, which were then subjected to a validation process. The time spent by the respondents on the entire survey was over 10 min and the time spent on viewing the manipulation message was over 10 s, which can ensure the validity of the data. Among these 217 respondents, 110 were females, 107 were males. They ranged in age from 18 to 50, with 67.34% clustered between 23 and 35. The majority of respondents have a college degree including bachelor's degree (49.77%) and master's degree and above (43.78%). Most (61.51%) of the respondents had an annual income greater than $5000, including 31.34% that had an annual income greater than $15000. Most (70.05%) of the respondents live in first-tier cities, including 11.98% in second-tier cities and 11.52% in third-tier cities in China. Conducted message intervention for one month, some respondents withdrew, who do not complete the reading of message materials or fill out the post-test questionnaire carefully, and there are 186 respondents who completed validly the whole experiment, which is shown in Table 2.

### 3.4. Analysis Procedures

All data were analyzed with SPSS 26.0. Descriptive statistical analysis, independent sample *t*-test, Scheffe posttest, and logistic binary regression were conducted to find out the important prediction and explanatory variables for the development of each stage of SCBF, and linear regression analysis to find out the important prediction and explanatory variables of SCBF in the action and maintenance stages, in order to find out the mediating variables of different framing-based green messages that have different effects on individuals at different stages of change.

## 4. Empirical Results

### 4.1. Reliability and Validity Analysis

SPSS 26.0 was used for reliability and validity tests in this study. The specific results are shown in Table 3. The interpretation rate of each variable reached the criterion of 70%, and the overall KMO value and Cronbach's *α* coefficient were 0.842 and 0.889, respectively, greater than 0.7. Meanwhile, the KMO (0.731–0.938) and Cronbach's *α* values (0.788–0.970) of each variable reached the acceptance standard 0.7. The measurement scale can be considered to be of good reliability and validity based on the above analysis.

### 4.2. Variables in Different Stages of SCBF

#### 4.2.1. Descriptive Statistical Analysis

Descriptive statistical analysis and variance analysis of the perceived benefits, perceived barriers, self-efficacy, and perceived threats were conducted to explore the changes of those variables in the process of SCBF and find out the important variables that explain the changes in each stage. The data collected through pretest questionnaire before the message intervention were used for analysis, and the results are shown in Table 4. The *F* value of perceived benefits is 14.703 (*p*=0.000 < 0.05), the *F* value of perceived barriers is 4.320 (*p*=0.006 < 0.05), the *F* value of self-efficacy is 28.457 (*p*=0.000 < 0.05), and the *F* value of perceived threats is 18.069 (*p*=0.000 < 0.05), which show that the mean values of each variable at different stages of SCFB are significantly different, indicating that there are significant differences in individual perceived interests, perceived barriers, self-efficacy, and perceived threats at different stages of SCBF. For convenience, the changes of SCBF are shown sequentially as phases in Table 4. Phase 1 represents the pre-intent phase, phase 2 the intent phase, phase 3 the preparation phase, and phase 4 the action and maintenance phase.

In order to more intuitively observe the changing trends of perceived benefits, perceived barriers, self-efficacy, and perceived threats at different stages of SCBF, the average values of each variable at different stages of SCBF are plotted, as shown in Figure 2. With the development of the changing stages of SCBF, the perceived benefits increase significantly in phase 1 to phase 2 and phase 3 to phase 4, with less increase in phase 2 to phase 3. In general, individual perceived benefits will keep increasing, perceived barriers will keep decreasing, self-efficacy will continue to increase with a large increase from phase 1 to phase 2 and from phase 3 to phase 4, and a smaller increase from phase 2 to phase 3, and perceived threats will continue to increase with gradually decreasing magnitude.

#### 4.2.2. Post Mortem Results

Scheffe method was used to conduct multiple comparisons for each variable changes in two phases to identify the stages in which the variables vary significantly. The results are shown in Table 5. It can be seen that in the formation of SCBF, adjacent changing stages with significant differences in perceived benefits are from phase 1 to phase 2 and phase 3 to phase 4 and perceived benefits are increased; in self-efficacy, they are from phase 3 to phase 4 and self-efficacy is increased; in perceived threats, they are from phase 1 to phase 2, and perceived threats are increased. There was no significant difference for perceived barriers in any changing stages.

#### 4.2.3. Logistic Regression Analysis

Logistic regression analysis was performed to determine the important prediction and explanatory variables when the adjacent change stage of SCBF is changed. First, the adjacent change stage is used as the dependent variable; the perceptual benefits, perceived barriers, self-efficacy, and perceived threats are selected into the equation for binary logistic regression analysis by the forward Wald method to get the important prediction and explanatory variables of moving forward of each adjacent change stages of SCBF. Then as phase 4 can no longer move forward, the linear regression analysis is used to obtain the important explanatory variables that remain unchanged after the behavior is formed. The logistic regression analysis results are shown in Table 6. It can be seen that perceived benefits and perceived threats can predict and explain the shift from phase 1 to phase 2, perceived threats can predict and explain the shift from phase 2 to phase 3, perceived benefits and self-efficacy can predict and explain the shift from phase 3 to phase 4, self-efficacy and perceived threats can predict and explain the maintenance of phase 4, and perceived threats play no role in the formation of SCBF. H6 was thus established.

### 4.3. Manipulation Check

The test value was set to 4 to ensure the effectiveness of the framing message control, and the single sample *t*-test was conducted to establish the manipulation test scale. The test results are shown in Table 7. *M* gain = 6.203 > 4, *t* = 24.592, *p*=0.000 < 0.05, and *M* loss = 6.333 > 4, *t* = 23.658, *p*=0.000 < 0.05, which demonstrated that the gain group and the loss group on the manipulation scale are significantly higher than 4 points and indicated that manipulation of the gain and loss framing messages is effective, the participants in the gain group and the loss group can distinguish the framing green messages they received, and the framing of experimental materials was obvious.

### 4.4. The Influence on Variables of the Green Message Framing at Different Stages of SCBF

The difference between the mean of the same score in the post-questionnaire and the pre-questionnaire was used to analyze the difference in the degree of change in the same variables of individuals at different stages of SCBF after receiving gain and loss framing messages. The independent sample *t*-test and univariate analysis in general linear models were used for comparison, and the results are shown in Table 8.

The difference in perceived threats was found to reach a significant level (*p*=0.005 < 0.05) in phase 1, indicating green messages from different framing on the changes in individual perception of threats were significantly different (*M* gain = 0.200, *M* loss = 3.267), the increase in perceived threats of individuals receiving loss framing messages was significantly higher than that of gain framing messages, and the effect value in this item was 0.247, which represents that there is a high correlation strength for differences between the framing messages and perceived threat changes. *R*^2^ is 0.220, indicating that the loss framing-based green messages can explain the 22.0% variation of the perceived threats. The results demonstrate that the loss framing-based green messages have a significant positive impact on the perceived threats in phase 1. Moreover, the above proves that the perceived threats are an important prediction and explanatory variable in SCFB from phase 1 to phase 2, so it is believed that loss framing-based green messages to enhance the individual's perceived threats are more conducive to the development of the change stages. H10a, H11a, and H12a were established.

The difference in perceived threats was found to reach a significant level (*p*=0.004 < 0.05) in phase1, indicating green messages from different framing on the changes in individual perception of threats were significantly different (*M* gain = −2.111, *M* loss = 1.647), the increase in perceived threats of individuals receiving loss framing messages was significantly higher than that of gain framing messages, and the effect value in this item was 0.221, which represents that there is a high correlation strength for differences between the framing messages and perceived threat changes. *R*^2^ is 0.197, indicating that the loss framing-based green messages can explain the 19.7% variation of the perceived threats. The results demonstrate that the loss framing-based green messages have a significant positive impact on the perceived threats in phase 2. Moreover, the above proves that the perceived threats are an important prediction and explanatory variable in SCFB from phase 2 to phase 3, so it is believed that loss framing-based green messages to enhance the individual's perceived threats are more conducive to the development of the change stages. H10b, H11b, and H12b were established.

The difference in perceived benefits was found to reach a significant level (*p*=0.009 < 0.05) in phase 3, indicating green messages from different framing on the changes in individual perception of benefits were significantly different (*M* gain = 2.000, *M* loss = −2.357, *p*=0.005 < 0.05), the increase in perceived benefits of individuals receiving gain framing messages was significantly higher than that of loss framing messages, and the effect value in this item was 0.233, which represents that there is a high correlation strength for differences between the framing messages and perceived benefit changes. *R*^2^ is 0.204, indicating that the gain framing-based green message can explain the 20.4% variation of the perceived benefits. The results demonstrate that the gain framing-based green messages have a significant positive impact on the perceived benefits in phase 3. Moreover, the above proves that the perceived benefits are an important prediction and explanatory variable in SCFB from phase 3 to phase 4, so it is believed that gain framing-based green messages to enhance the individual's perceived benefits are more conducive to the development of the change stages. H7a, H8a, and H9a were established. Furthermore, the difference in self-efficacy was found not to reach a significant level (*p*=0.695 < 0.05) in phase 3, indicating there is no significant difference for green messages from different framing on the changes in individual self-efficacy. H3a, H4a, and H5a were not established. This may be because the individuals have not yet carried out SCBF in phase 3, and they need to be surrounded by more tips and guidance related to SCBF, so that the improvement of self-confidence is not enough to promote the development of their behavior.

The differences in perceived benefits (*p*=0.000 < 0.05) and self-efficacy (*p*=0.004 < 0.05) were found to reach a significant level in phase 4, indicating green messages from different framing on the changes in individual perceived benefits (*M* gain = 2.941, *M* loss = −1.353) and self-efficacy (*M* gain = 3.235, *M* loss = −2.353) were significantly different, the increase in perceived benefits and self-efficacy of individuals receiving gain framing messages was significantly higher than that of loss framing messages, and the effect value *η*^2^ in the items was 0.367 and 0.236, which represent that there is a high correlation strength for differences between the framing messages and perceived benefit and self-efficacy changes. *R*^2^ is 0.347 and 0.212, indicating that the gain framing-based green messages can explain the 34.7% variation of the perceived benefits and 21.2% variation of the self-efficacy. The results demonstrate that the gain framing-based green messages have a significant positive impact on the perceived benefits and self-efficacy in phase 4. Moreover, the above proves that self-efficacy is an important prediction and explanatory variable in SCFB from phase 4, while perceived benefits are not, so it is believed that gain framing-based green messages to enhance the individual's self-efficacy are more favorable to stay in phase 4 for them. H3b, H4b, H5b, and H7b were established and H8b and H9b were not established. This may be because consumers in phase 4 have been more familiar with SCBF, and they can perceive benefits conveyed by the gain framing-based green messages, but they have their own judgment on whether these benefits can really come true, so they will not maintain the current behavior based on their perceived benefits.

### 4.5. The Effects of the Green Message Framing on Individuals at Different Stages of SCBF

The blank group without any green message framing was designed to further demonstrate the effect of green message framing on the formation of SCBF. The differences between the change stages before and after the message framing were compared by the Wilcoxon symbolic rank and test of the paired samples, and the outcome differences between loss group and blank group after message framing intervention were compared as shown in Table 9. Subsequently, the independent sample Mann–Whitney *U* test was used to further compare the degree of stage changes between loss group and blank group.

Before the loss framing intervention, there are 15 people in loss group and blank group in the pre-intention stage, and 7 people in loss group entered the intention stage, 4 people entered the preparation stage, 2 people entered the action and maintenance stage, and the remaining 2 people did not change, and the change was significant (*p*=0.001 < 0.05) after loss framing intervention. At the same time, 2 people in blank group entered the intention stage, the remaining 13 people did not change, and there was no significant difference in the change (*p*=0.157 < 0.05). In addition, the results show a significant difference (*p*=0.000 < 0.05) for the stage changes between loss group and blank group, which indicates that loss framing effect is significantly better toward the formation of SCBF in phase 1 than that of blank group.

Before the loss framing intervention, there are 17 people in loss group in the intention stage, and 4 people in loss group entered the preparation stage, 11 people entered the action and maintenance stage, and the remaining 2 people did not change, and the change was significant (*p*=0.000 < 0.05). At the same time, 15 people in blank group were in the intention stage, 1 person in blank group entered the preparation stage, 4 people entered the action and maintenance stage, 3 people retreated to the pre-intention stage, and the remaining 7 people did not change, and there was no significant difference in the change (*p*=0.132 < 0.05) after loss framing intervention. In addition, the results show a significant difference (*p*=0.004 < 0.05) for the stage changes between loss group and blank group, which indicates that loss framing effect is significantly better toward the formation of SCBF in phase 2 than that of blank group.

Before the gain framing intervention, there are 14 people in gain group and blank group in the preparation stage, and 11 people in gain group entered the action and maintenance stage, and the remaining 3 people did not change, and the change was significant (*p*=0.001 < 0.05). At the same time, 3 people in blank group entered the action and maintenance stage, 3 people retreated to the intention stage, and the remaining 7 people did not change, and there was no significant difference in the change (*p*=0.527 < 0.05) after gain framing intervention. In addition, the results show a significant difference (*p*=0.002 < 0.05) for the stage changes between gain group and blank group, which indicates that gain framing effect is significantly better toward the formation of SCBF in phase 3 than that of blank group.

Before the gain framing intervention, there are 17 people in gain group in the action and maintenance stage, and the remaining 17 people did not change, and the change was not significant (*p*=1.000 < 0.05). At the same time, 15 people in blank group entered the action and maintenance stage, 1 person retreated to the intention stage, 1 person retreated to the pre-intention stage, and the remaining 13 people did not change, and there was no significant difference in the change (*p*=0.180 > 0.05) after gain framing intervention. In addition, the results show no significant difference (*p*=0.126 > 0.05) for the stage changes between gain group and blank group, which indicates that gain framing effect has higher behavior stability toward SCBF in phase 4 than that of blank group.

## 5. Discussion and Conclusion

### 5.1. Theoretical Implications

The impact of green messages on consumer environmental behavior has been widely confirmed, and the influence of green message framing on individual environmental behavior has been proved. There are many different ways to divide the green message framing, but the benefit and loss framing, as one of the important frameworks for promoting consumer decision making, has not yet been agreed. Therefore, this article frames the benefits and losses of green messages, aims to explore the impact mechanism of green message framing on the SCBF, and provides suggestions for enterprises to carry out more targeted green marketing. Furthermore, the cross-theoretical model can comprehensively explain the behavior change of individuals through four parts including change stage, change process, decision balance, and self-efficacy, which not only pays attention to why behavior changes, but also pays attention to how behavior changes. The application of cross-theoretical models in the field of healthy behaviors has been very mature, and the applicability in the field of sustainable consumer behavior has been proven.

Communicating the need for sustainable consumption and presenting new related policy initiatives require a good understanding of how the public are motivated to be sustainable. This study examined how gain and loss framing-based green messages influenced participants' changing stages in SCBF and perceived outcome benefits, barriers, efficacy, and threats related to SCBF and, more importantly, how individual differences in perceived benefits, perceived barriers, self-efficacy, and perceived threats interacted with these framing manipulations. This study yielded several findings of interest which, we believe, underscore the importance of considering the perceived outcome and predisposition of an individual when framing green messages about the formation of SCBF.

Theoretically, this study contributed to the description of the framing of green messages in the formation of SCBF. We found that effects of framing green messages on the formation of SCBF will vary depending on the change stage that individuals are in. In the pre-intention stage and the intention stage, the SCBF is mainly because the loss framing-based green message promotes the improvement of individual perceived threats. The SCBF in the preparation stage and the action and maintenance stage is mainly due to the fact that the gain framing-based green message promotes the improvement of perceived benefits in individual self-efficacy and decision balancing.

Another contribution is the introduction of transtheoretical model into the field of sustainable fashion consumption behavior. It constructs and verifies the theoretical model of gain and loss framing of green messages and the four changing stages of SCBF and explains the intrinsic mechanism of “intention-behavior” of SCBF. Results imply that perceived benefits and perceived threats may be a more tangible outcome of SCBF for many people; the perception on green message framing should not be ignored and may be a more significant driver for SCBF. This study provides new ideas for the follow-up studies of SCBF and provides references for enterprises to formulate more effective green messages intervention strategies.

Our study also points to the value of intervention strategies of green messages to reduce the gap of “intention-behavior” in SCBF, because results show that green messages have a framing effect in the formation of SCBF, and individuals at different changing stages react differently after receiving different framing green messages. Loss framing can significantly promote the development of individual behaviors in phase 1 and phase 2, while gain framing can significantly promote the development of individual behavior in phase 3 and maintain the stability of individual behaviors in phase 4. Furthermore, the effects of green message framing are different for each phase. In phase 1 and phase 2, the difference in changes between gain group and loss group reaches a significant level in terms of perceived threats including greater change in loss group, and perceived threat is an important prediction and explanatory variable for SCBF from phase 1 to phase 2 and from phase 2 to phase 3, thus loss framing green messages should be more conductive to the moving forward of changing stage in SCBF. In phase 3, the difference in changes between gain group and loss group reaches a significant level in terms of perceived benefits including greater change in gain group, and perceived benefit is an important prediction and explanatory variable for SCBF from phase 3 to phase 4, thus gain framing green messages are more conducive to the development of individual behavior. In phase 4, the difference in changes between gain group and loss group reaches a significant level in terms of perceived benefits and self-efficacy including greater change in gain group, and self-efficacy is an important prediction and explanatory variable for SCBF to maintain in phase 4, thus gain framing green messages can enhance self-efficacy to promote the maintenance of SCBF.

### 5.2. Practical Implications

In an era of increasing concern about environment and resources, insights into consumers' adoption of SCBF will have applications for fashion enterprises to carry out green marketing and promote SCBF. Findings demonstrate that green message framing effects were observed when consumers received positive or negative green messages. The implication is that participants at different changing stages of SCBF are likely to perceive green messages in quite different ways from each other. There is therefore unlikely to be a same message that can effectively engage everyone. The reasons why the differences in “intention-behavior” of sustainable consumption of fashion became salient for some of our participants to a greater extent than others remain unexplained and potential individual perception differences that may explain why expression differences of green messages have affected people differently should be explored further [39]. For example, people who already have sustainable consumption intention may be more likely to be influenced by engaging with loss-framed green messages, and people who already have sustainable consumption behavior may be more likely to be influenced by engaging with gain-framed green messages.

Overall, we find green message framing is useful in engaging people with SCBF and could result in greater levels of SCBF given the outcomes of our perceptions. This finding highlights the importance of considering and accounting for the potential of behavioral changes in the potential impact of expression of green message displays.

Based on the findings in this study, enterprises may need to place more managerial and marketing efforts into consumers' perception on green messages framing. When exposed to effective green messages, consumers may change their intention and behavior toward SCBF so that they can make contribution to promoting green marketing and protecting the environment [44]. In addition, the fashion enterprises also need to identify what changing stages that individuals are in and what motivates individuals to change their intention or behavior of SCBF. The enterprises could promote and enhance green fashion marketing, actively establish a green brand image, and take the initiative to assume the responsibility of protecting the environment because consumer demands for green fashion products and services were realized, which they believed to save resources and protect the environment through SCBF.

Finally, it is worth mentioning that green messages are important means of disseminating green ideas, and contact with more green messages may greatly affect consumers' understanding of environmental issues, correct their misconceptions about fashion consumption, and then stimulate their determination to carry out sustainable consumption as well as take the initiative to understand SCBF, inspire themselves to change SCBF, and ultimately achieve sustainable consumption behavior. In this way, consumers may save resources and reduce waste through SCBF, improving the ecological environment and thus the quality of life. Meanwhile, consumers' demand for green products will increase, thus prompting enterprises to change traditional production methods, actively establish a green brand image, and take the initiative to assume the responsibility of protecting the environment. Obviously, in order to alleviate the pollution problem of the garment industry, it is the key means to promote the formation of SCBF.

### 5.3. Limitations and Future Research Avenues

Our results are limited by the use of young people aged from 18 to 25 within this study and therefore the generalizability of our results is limited. However, this sample was homogenous across conditions, giving assurance to the reliability of results noted. In addition, given that a young and well-educated sample is already likely to be more environmentally concerned, we should suggest that the observed green message framing effects might be stronger in a broader cross-section of the population. Further, the message intervention experiment and questionnaire survey were conducted online throughout the process, which may not help in understanding the real situation of the respondents, and some respondents didn't finish the whole experiment, resulting in an unstable number of experimental samples. Therefore, future research is recommended to focus on these topics in order to combine online and offline methods to ensure that participants take each experiment seriously and do not quit halfway.

When perceived benefits or perceived threats are salient within either a particular context or social group, then our findings suggest that this might in itself be enough to promote sustainable fashion consumption behaviors. Thus, in the development of an efficient green message intervention strategy, besides the gain and loss framing green messages, individuals' uniqueness and self-efficacy decision making have also to be taken into account to further generalize the conclusions to a wider range of applications. In addition, the psychology and behavior of consumers can also be tested using neural mechanism-related methods, so that the experimental results are more realistic and reliable.

## Figures and Tables

**Figure 1:** Cross-theoretical model.

**Figure 2:** Changes of variables in different stages of SCBF.

**Table 1:** Green message intervention schedule.

Number of interventions	Day
Intervention 1	1
Intervention 2	3
Intervention 3	5
Intervention 4	7
Intervention 5	10
Intervention 6	14
Intervention 7	18
Intervention 8	24
Intervention 9	30

**Table 2:** Number of respondents at different stages of change in each experimental group.

	Preintention	Intention	Preparation	Action and maintenance	Total
Gain framing group	15	18	14	17	64
Loss framing group	15	17	14	17	63
Blank group	15	15	14	15	59
Total	45	50	42	49	186

**Table 3:** Reliability and validity analysis.

Variables		Cronbach's *α*	KMO	Interpretation rate (%)
Decision balancing	Perceived benefits	0.970	0.822	82.20
	Perceived barriers	0.866		

Self-efficacy		0.917	0.880	75.58
Perceived threats		0.731	0.731	83.61

Dependent variables	Preintention stage	0.788	0.938	78.08
	Intention stage	0.952		
	Preparation	0.927		
	Action and maintenance stage	0.959		

**Table 4:** Descriptive statistics of variables in different change stages of SCBF.

Variables	Phase 1	Phase 2	Phase 3	Phase 4	*F* value	*P* value
Perceived benefits	5.420 ± 1.071	5.952 ± 0.887	6.006 ± 0.829	6.476 ± 0.9690	14.703^*∗*^	≤0.001
Perceived barriers	4.686 ± 0.884	4.365 ± 0.988	4.205 ± 0.846	4.017 ± 1.202	4.320^*∗*^	0.006
Self-efficacy	4.068 ± 0.906	4.542 ± 0.786	4.718 ± 0.739	5.457 ± 0.898	28.457^*∗*^	≤0.001
Perceived threats	4.007 ± 1.338	4.891 ± 0.887	5.311 ± 0.896	5.446 ± 1.179	18.069^*∗*^	≤0.001

Note: ^*∗*^*P* is significant below 0.05.

**Table 5:** Comparison of differences of variables in change stages of SCBF.

Variables	(*I*) Change stages	(*J*) Change stages	Mean difference (*I*-*J*)	Stand deviation	*P* value
Perceived benefits	1	2	−0.531^*∗*^	0.173	0.026
		3	−0.585^*∗*^	0.180	0.016
		4	−1.032^*∗*^	0.160	≤0.001
	2	3	−0.054	0.176	0.993
		4	−0.501^*∗*^	0.155	0.017
	3	4	−0.470^*∗*^	0.164	0.043

Perceived barriers	1	2	0.321	0.205	0.488
		3	0.482	0.214	0.171
		4	0.669^*∗*^	0.190	0.007
	2	3	0.161	0.209	0.898
		4	0.348	0.185	0.316
	3	4	0.188	0.194	0.818

Self-efficacy	1	2	−0.474	0.170	0.053
		3	−0.650^*∗*^	0.177	0.004
		4	−1.389^*∗*^	0.157	≤0.001
	2	3	−0.176	0.173	0.793
		4	−0.914^*∗*^	0.153	≤0.001
	3	4	−0.739^*∗*^	0.161	≤0.001

Perceived threats	1	2	−0.884^*∗*^	0.222	0.002
		3	−1.304^*∗*^	0.231	≤0.001
		4	−1.439^*∗*^	0.205	≤0.001
	2	3	−.0420	0.226	0.329
		4	−0.555	0.199	0.054
	3	4	−0.135	0.210	0.937

Note: ^*∗*^*P* is significant below 0.05.

**Table 6:** Regression results of variables between adjacent change stages of SCBF.

Logistic regression equation	*P* value	
*Y* (phase 1 − phase 2) = 0.755*∗*perceived benefits + 0.514*∗*perceived threats − 6.465	Perceived benefits	0.010
	Perceived threats	0.032

*Y* (phase 2 − phase 3) = 0.541*∗*perceived threats − 2.926	Perceived threats	0.028

*Y* (phase 3 − phase 4) = 0.641*∗*perceived benefits + 0.807*∗*self-efficacy − 7.496	Perceived benefits	0.026
	Self-efficacy	0.004

*Y* (phase 4) = 0.685*∗*self-efficacy + 0.188*∗*perceived threats	Self-efficacy	≤0.001
	Perceived threats	0.020

Note: ^*∗*^*P* is significant below 0.05.

**Table 7:** Experimental maneuverability test results.

	Number of cases	*t*	DF	Sig.	Mean	Standard deviation	95% confidence interval	
							Lower limit	Upper limit
Gain framing group	64	24.592	63	0.000	6.203	0.72	2.0241	2.3821
Loss framing group	63	23.657	62	0.000	6.333	0.78	2.1362	2.5305

**Table 8:** Comparison of the changes of variables in SCBF for gain group and loss group.

	Group	No. of cases	Mean	SD	*p*	*t*	*η* ^2^	*R* ^2^
Phase 1								
Perceived threats	Gain framing	15	0.200	2.651	0.005	−3.028	0.247	0.220
	Loss framing	15	3.267	2.890				

Phase 2								
Perceived threats	Gain framing	18	−2.111	3.376	0.004	−3.058	0.221	0.197
	Loss framing	17	1.647	3.888				

Phase 3								
Perceived benefits	Gain framing	14	2.000	4.132	0.009	2.811	0.233	0.204
	Loss framing	14	−2.357	4.069				
Self-efficacy	Gain framing	14	2.786	4.371	0.695	0.397		
	Loss framing	14	2.000	5.974				

Phase 4								
Perceived threats	Gain framing	17	2.941	2.968	0.000	−4.303	0.367	0.347
	Loss framing	17	−1.353	2.849				
Self-efficacy	Gain framing	17	3.235	3.898	0.004	−3.145	0.236	0.212
	Loss framing	17	−2.353	6.204				

Note: *η*^2^ ≥ 0.14 indicates that there is high correlation between the grouping variable and the test variable, 0.14 > *η*^2^ > 0.06 indicates moderate correlation, and *η*^2^ ≤ 0.06 indicates low correlation.

**Table 9:** Changes of different stages of the framing group and the blank group.

Group	Changes of different stages of SCBF				*Z*	*P* value
	Phase 1	Phase 2	Phase 3	Phase 1		
Phase 1						
Loss framing	2	7	4	2	−3.247^b^	0.001
Blank	13	2	0	0	−1.414^b^	0.157

Phase 2						
Loss framing	0	2	4	11	−3.578^b^	≤0.001
Blank	3	7	1	4	−1.508^b^	0.132

Phase 3						
Gain framing	0	0	3	11	−3.317^b^	0.001
Blank	1	3	7	3	−0.632^c^	0.527

Phase 4						
Gain framing	0	0	0	17	−0.000^b^	1.000
Blank	1	1	0	13	−1.342^b^	0.180

## Data Availability

The data can be provided by the corresponding author on request.
